# Application of Nursing Intervention Plan Based on Symptom Management Theory among Breast Cancer Patients

**DOI:** 10.1155/2022/3816768

**Published:** 2022-08-18

**Authors:** Qingqing Xu, Yu Chen, Xiaping Shen, Qunying Fang

**Affiliations:** ^1^Department of Thyroid and Breast Surgery, Zhejiang Xiaoshan Hospital, Zhejiang, Hangzhou 311201, China; ^2^Department of Breast Surgery, Cancer Hospital of The University of Chinese Academy of Sciences, Zhejiang, Hangzhou 310022, China

## Abstract

In order to explore the application effect of nursing intervention based on symptom management theory in breast cancer patients, a total of 120 breast cancer patients who were hospitalized in the Thyroid and Breast Surgery Department of Zhejiang Xiaoshan Hospital from July 2018 to July 2021 were selected as the research subjects. Patients from the control group received routine nursing, while patients from the intervention group underwent nursing interventions based on symptom management theory. Before and after the intervention, symptom distress, Herth Hope Index, quality of life, self-rating anxiety scale (SAS), self-rating depression scale (SDS), visual analogue score (VAS), and Pittsburgh sleep quality index (PSQI) were evaluated in two groups. The results showed that the symptom severity score and the symptom distress score, SAS scores, SDS scores, VAS scores, and PSQI scores in the intervention group were significantly lower than those in the control group, while the Herth Hope Index scores and FACT-B scores in the intervention group were obviously higher than those in the control group (all *P* < 0.05) after intervention. In conclusion, nursing interventions based on symptom management theory could decrease symptom distress among breast cancer patients, increase their hope levels, improve their life quality, relieve the negative emotions, enhance the sleep quality, and reduce their pain. It is worthy of clinical application.

## 1. Introduction

Breast cancer is one of the most common malignant tumors in women, and its incidence accounts for 7–10% of all malignant tumors in the whole body. Its incidence is often related to heredity, and between the ages of 40 and 60, the incidence of women before and after menopause is higher. It is one of the most common malignant tumors that usually occurs in the glandular epithelium of the breast, seriously affecting women's physical and mental health and even life-threatening. Chemotherapy refers to the use of drugs to treat a disease. Surgery and radiation kill cancer cells in specific areas, while chemotherapy works throughout the body. Chemotherapy can destroy cancer cells that have spread to various parts of the body. With the emergence of new drugs and the strengthening of the status of chemotherapy in recent years, the cure rate of breast cancer has been significantly improved. However, chemotherapy has its own shortcomings, mainly because the side effects are too large, which is difficult for patients to accept [1]. However, chemotherapeutic drugs could kill the tumor cells and simultaneously damage normal cells to a certain extent and have an inhibitory effect on immune function. Patients with breast cancers usually have corresponding psychological and physiological symptoms following the chemotherapy. Psychological symptoms manifested as anxiety, intensive concentration, depression, and other emotions [2–4], while physiological symptoms often showed vomiting, fatigue, weight reduction, cachexia, alopecia, and so on, and a few cases showed decreased libido and neurological signs. In different stages of treatment for these breast cancer patients, adverse physiological reactions and heavy psychological burden would make patients to be unable to coordinate treatment, ultimately affecting the life quality and healing process [5, 6]. Therefore, how to improve the symptoms of breast cancer patients during the period of treatment, help patients increase the life quality and recuperate as soon as possible and return to society have become the key issue of current research.

Symptom management theory (SMT) is developed from the symptom management model (SMM) of the University of California at San Francisco School, which describes symptom management as a multidimensional process [7]. In SMM, symptom management is composed of three interactive parts: symptom experience, symptom management strategies, and outcomes [8]. SMM assumes that effective symptom management needs to take all three parts into account. Larson et al [3] reported that SMT was considered as the middle-range theories (MRTs), and individualized intervention was performed through the evaluation of patients' clinical symptoms, which could significantly improve the patients' discomfort and emotional state and increase the life quality. At present, SMT is widely used in clinical practices and scientific research, and has been extensively studied in various adult diseases such as diabetes, heart disease, chronic lung disease, chronic pain, and cancer, and has achieved good results [9–11]. Kanungpairn et al. reported that a symptom management program could attenuate auditory hallucinations in outpatients diagnosed with schizophrenia through their understanding of symptoms and learning and practicing skills for managing their symptoms [12]. A detailed analysis of SMT along with its application in adult cancer in 20 oncology research studies showed SMT could provide useful guidance for adult oncology research and nursing practices [10]. However, there have been no relevant reports on the application effects of the intervention model based on SMT among breast cancer patients. Whether SMT applications could affect the recovery effects in breast cancer patients needs further research.

In this study, a total of 120 patients with breast cancer who were hospitalized in the Department of Thyroid and Breast Surgery of Zhejiang Xiaoshan Hospital from July 2018 to July 2021 were selected as the research subjects. The patients were randomly divided into a control group and an intervention group, with a total of 60 cases in each group. Herth Hope Index, the scores of symptom severity and symptom distress, life quality scores, self-rating anxiety scale (SAS), self-rating depression scale (SDS), Pittsburgh sleep quality index (PSQI), and visual analogue score (VAS) were used as the major observations. The results of this study would provide a scientific basis for clinical nursing measures in breast cancer patients.

## 2. Materials and Methods

### 2.1. Subjects

In this study, 120 breast cancer patients admitted into the Department of Thyroid and Breast Surgery in Zhejiang Xiaoshan Hospital from June July 2018 to July 2021 were enrolled using the convenience sampling method. Inclusion criteria: (1) Female; (2) Over 18-years old; (3) patients were clinically diagnosed as breast cancer; (4) patients received chemotherapy and 12 weeks follow-up were completed; (5) patients were not diagnosed with spirit system disease before admission and able to communicate normally with investigators; (6) patients had a detailed understanding of the content of this study and obtained informed consent before participating; (7) patients were able to exploit the WeChat application. Exclusion criteria: (1) Patients had a disease that seriously affected their own health before the participation; (2) patients had different degrees of cognitive impairment and could not understand various nursing operations.

According to the inclusion and exclusion criteria, 120 patients with breast cancer were enrolled in this retrospective study. For the control group, 60 patients received routine nursing intervention. For the intervention group, 60 patients were treated with a nursing care model based on symptom management theory. This study was approved by the Ethics Committee of Zhejiang Xiaoshan Hospital and informed consent was signed by these patients.

### 2.2. Methods

Patients in the control group were treated with routine nursing. In this group, routine admission education and health education were performed. Good nursing work for the perioperative period of breast cancer was done. Discharge education was also conducted on discharge from the hospital, which included home-based rehabilitation and announcements for reexamination. Pay attention to observing the emotions in patients. Psychological counseling was done well, and the methods and skills of psychological regulation were guided for patients.

Patients in the intervention group received a nursing care model based on symptom management theory besides routine nursing. The intervention time was from the admission to 3 months after hospital discharge. This group consists of a nursing intervention team consisting of a head nurse, 4 junior nurses, 1 doctor, and 1 psychological counselor. Each member has at least 5 years of breast cancer work experience and is more than an intermediate technical title. The head nurse is responsible for the organization and management of the entire project. The doctor was responsible for the treatment and condition monitoring of the patients. The nurses and psychological consultant were specifically responsible for the implementation of nursing interventions in patients. All of the members of this team had undergone systematic and professional training and held qualification certificates before their interventions were performed on patients.

The details regarding nursing care plans based on symptom management theory were as follows: ① Evaluation of symptom experience in breast patients were performed. The Chinese version of the Memory Symptom Evaluation Scale [13] was used to conduct a preliminary evaluation on 60 patients by a full-time nurse. This questionnaire was mainly used for the evaluation of physical and psychological symptoms in patients with malignant tumors. It was composed of 32 items such as pain-related symptom clusters, psychological symptom clusters, perimenopausal symptom clusters, gastrointestinal-related symptom clusters, neurological-related symptom clusters, and impaired self-image symptom clusters. The 24 items from the first part were used for evaluating symptoms during treatment in terms of four domains such as incidence, frequency, severity, and distress, while the 8 items from the second part were applied for evaluating symptoms in terms of three dimensions such as incidence, severity, and distress. The degree of frequency was scored as 1 point (rarely), 2 points (sometimes), 3 points (frequently) and 4 points (continuously). The degree of severity was scored as 1 point (mild), 2 points (moderate), 3 points (severe) and 4 (very severe). The level of distress was scored as 0 point (none), 1 points (a little), 2 points (some), 3 points (more) and 4 points (a lot), respectively. ② According to the scoring rules of the questionnaire, the average scores for the degree of frequency, severity, and distress in terms of symptoms were considered the symptom scores. For symptoms with only severity and distress scores, the average score in terms of these two aspects was defined as the symptom scores. According to the results of the evaluation, the major symptom cluster scores for breast cancer patients following chemotherapy are shown in Table 1. ③ Symptom management strategies: According to the evaluation results of symptom experience in patients, items such as current symptoms, the frequency and severity of symptoms, whether to use drug therapy, whether to use nonmedicine intervention, and so on were assessed. The corresponding nursing intervention plan was formed. The interventions were performed by requiring, participating, and conferring, respectively.

The required intervention was performed for patients with self-image damaged symptom clusters and perimenopausal symptom clusters. Patients were required to participate. The nurse gave the patients a face-to-face interview, encouraged the patients to tell the changes in their bodies after chemotherapy, and asked ”do you feel tired”, “do you need to rest,” “what kind of relaxation do you feel you need,” etc. Understand the needs of self-image impaired symptoms and perimenopausal symptoms faced by patients and meet their needs to the greatest extent. Inform patients that the impact of chemotherapy on their self-image was an experience in recovery, and that it could bring more things and insights besides the disease itself. They could not choose to escape and resist and were informed that they should accept as much as possible. And if they try to control their own feelings, it may be worse. Instruct patients to keep a daily diary to record how they feel about symptoms. The intervention measures, such as aerobic exercise and music therapy were performed to relieve perimenopausal symptoms in patients. For patients with gastrointestinal symptom clusters and pain-related symptom clusters, the intervention team arranged the follow-up visits according to the needs of the patients. The patients were evaluated in terms of physiology, psychology, and behavior. Further guidance on the treatment of side effects of chemotherapy, medication, diet, exercise, etc., was provided. The intervention team would receive timely information or feedback and propose improvement to the plans. Patients were encouraged to participate in an experience sharing session once a week to share their experiences in the face of nausea, vomiting, weight loss, pain, abdominal distension, and dizziness, and to help patients arrange some relaxation activities and rest, so that they could gradually form good living habits. For patients with mental symptom clusters and nervous system-related symptom clusters, the conferring intervention was provided due to low degree of symptoms. Give patients full trust and understanding and provide them with deeper levels of health knowledge. The patients should follow the WeChat official account. The WeChat official account automatically pushes a piece of popular science knowledge every day, as well as the content involved in the methods to relieve mental tension, sadness, anxiety, dizziness, numbness of hands and feet, and other symptoms. Patients should click to express their understanding or incomprehension after reading it. When patients cannot understand the knowledge points, the nurses should timely provide individual counseling in the form of voice, text, or video through the WeChat official account. Moreover, the team also should evaluate the effect and improvement of disease symptom management and whether there were noncompliance behaviors and their reasons, and discuss the solutions to the noncompliance behaviors with patients and allow the patients to give feedback on their own symptom management and treatment, drugs, and other adverse reactions. The satisfaction of intervention plans and their results from patients and their families were assessed. The team should evaluate whether the intervention plan had any side effects, discuss the possible reasons for not achieving the expected goals with patients, and formulate the next expected goals. The next step program of diagnosis, treatment, and medicine should also be provided.

### 2.3. Outcome Measures

#### 2.3.1. Symptom Distress

The Chinese version of the Anderson Symptom Assessment Scale (MDA-SI) was used to evaluate the symptom distress in both groups after intervention. It included the symptom severity scores and symptom distress scores. The symptom severity score was composed of 13 items such as pain, fatigue, nausea, disturbed sleep, shortness of breath, and forgetfulness. The symptom distress score included 6 items such as mood, general activities, work, and social relations. The scale was from 0 to 10 points. The symptom severity score was positively correlated with the severity of symptoms, while the symptom distress score was positively associated with the degree of distress caused by symptoms affecting daily life.

#### 2.3.2. Herth Hope Index

The level of hope in patients before and after intervention was evaluated through the Herth Hope Index. It measured three dimensions in terms of the positive attitude towards the future and present, taking positive actions, and maintaining close relationships with others. The questionnaire consisted of 12 items responded to on a four-point Likert-type scale, scored as 1 (absolutely disagree), 2 (disagree), 3 (agree), and 4 (absolutely agree) [14]. The total score of this questionnaire varies from 12 to 48. Higher scores indicated a better hopefulness status.

#### 2.3.3. Quality of Life

The Chinese version of the Function Assessment of Cancer Therapy-Breast (FACT-B) was used to evaluate the quality of life in patients with breast cancer [15]. It was composed of five domains such as physical well-being, social/family well-being, emotional well-being, functional well-being, and additional concerns. This questionnaire included 36 items, and each item was scored according to a four-point scale. The high scores indicated a better quality of life.

#### 2.3.4. Negative Emotions

The self-rating anxiety scale (SAS) and self-rating depression scale (SDS) were used to assess the negative emotions in breast cancer patients. Both SAS and SDS included 20 items scored by a 4-point method. The higher score indicated the severity of anxiety and depression.

#### 2.3.5. Evaluation of Pain

The visual analogue score (VAS) was applied for evaluating the pain degree before and after intervention. The total score was 10 points. Higher scores suggested more pain.

#### 2.3.6. Quality of Sleep

Pittsburgh sleep quality index (PSQI) was used for assessing the sleep quality. It included 7 domains in the term of 18 items. The total score was21 points. Less than 7 scores indicated basic satisfaction with sleep quality, and more than 7 scores suggested poor quality of sleep.

### 2.4. Statistical Methods

The data included in this study were analyzed using SPSS statistical software version 19.0 (IBM, USA). The measurement data were calculated as the mean ± standard deviation. Independent-samples *T* test was applied for the comparison between two groups, while paired *t*-test was used for before-after comparison within the same group. The enumeration data were presented as number/percentage (*n*/%). A chi-square test was used for comparison between the two groups. *P* < 0.05 suggested statistically significant differences.

## 3. Results

### 3.1. Basic Data

As displayed in Table 2, there were no significant differences concerning age, degree of education, duration of the disease, BMI, neoplasm staging, marriage status, health insurance, job, and underlying diseases between the two groups (all *P* > 0.05) and they were comparable.

### 3.2. Comparison of Symptom Distress

As shown in Table 3, there were no significant differences regarding the symptom severity score and the symptom distress score before intervention between the two groups (7.2 ± 2.2 vs 7.0 ± 2.4, *P* > 0.05) (8.2 ± 2.0 vs 8.0 ± 1.8, *P* > 0.05). The symptom severity score and the symptom distress score in two groups after intervention were significantly decreased when compared with those before intervention (both *P* < 0.05). Compared with the control group, the symptom severity score and the symptom distress score after intervention were significantly lower in the intervention group (6.3 ± 2.0 vs 5.4 ± 2.1, *P* < 0.05; 6.4 ± 1.8 vs 5.5 ± 2.0, *P* < 0.05).

### 3.3. Comparison of Herth Hope Index

Before the intervention, there was no significant difference in the Herth Hope Index in terms of three dimensions between the two groups. After the intervention, the scores of both groups were significantly increased (all *P* < 0.05), while the scores of the Herth Hope Index in the intervention group were significantly more than those in the control group (all *P* < 0.05), as shown in Table 4. For example, before the intervention, there was no significant difference between the control group's positive attitude score of 9.0 and the intervention group's 9.3, but after the intervention, the control group had a positive attitude score of 10.4 and the intervention group was 12.2, and a significant difference was achieved between the two groups. The same is true for the other two indicators. These data show that nursing intervention programs based on symptom management theory meet the needs of breast cancer patients receiving chemotherapy and can effectively improve symptomatic distress.

### 3.4. Comparison of Life Quality

Before the intervention, there was no significant difference in life quality scores. After the intervention, the scores of the two groups significantly increased (*P* < 0.05), while the scores of physical well-being, social/family well-being, emotional well-being, functional well-being, additional concerns, and the mean scores in the intervention group were much higher than those in the control group (all *P* < 0.001), as shown in Table 5.

### 3.5. Comparison of SAS and SDS Scores

As shown in Figure 1, there were no obvious differences regarding SAS and SDS scores between the two groups before intervention (59.6 ± 4.7 vs 58.4 ± 4.2, *P* > 0.05; 55.9 ± 3.8 vs 56.3 ± 4.0, *P* > 0.05); SAS and SDS scores were obviously reduced in the intervention group after intervention when compared with those before intervention (both *P* < 0.05); Compared with the control group, SAS and SDS scores were obviously less than those in the intervention group after intervention (58.0 ± 3.9 vs 41.8 ± 3.5, *P* < 0.05; 53.8 ± 3.1 vs 37.6 ± 2.5, *P* < 0.05). These experimental results show that nursing intervention based on symptom management theory can effectively alleviate the symptoms of breast cancer patients, reduce patient anxiety, and improve the patient's life well-being index.

### 3.6. Comparison of VAS and PSQI Scores

A visual analogue scale (VAS) was used for pain assessment. It is widely used clinically in China. The basic method is to use a walking scale about 10 cm long. One side is marked with 10 scales, and the two ends are respectively “0” and “10.” A score of 0 means no pain. A score of 10 represents the most excruciating pain. The Pittsburgh Sleep Quality Index (PSQI) is suitable for the evaluation of sleep quality in patients with sleep disorders and mental disorders, as well as for the evaluation of sleep quality in the general population. The total score ranges from 0 to 2l, with higher scores indicating poorer sleep quality. As seen in Figure 2, the statistical differences were not found in terms of VAS scores (5.3 ± 0.8 vs 5.2 ± 0.6, *P* > 0.05) and PSQI scores (7.6 ± 0.9 vs 7.5 ± 0.8, *P* > 0.05) before intervention between the two groups. In the intervention group, VAS scores and PSQI scores after intervention were significantly lower than those before intervention. Compared with the control group, VAS scores and PSQI scores after intervention in the intervention group were significantly decreased (5.0 ± 0.7 vs 3.0 ± 0.4, *P* < 0.05; 7.4 ± 0.7 vs 4.8 ± 0.5, *P* < 0.05). These experimental results suggest that nursing interventions can improve symptoms in breast cancer patients.

## 4. Discussion

The treatment methods for breast cancer mainly included surgery, radiotherapy, and chemotherapy. With the continuous development of treatment methods, the recurrence risk and mortality of breast cancer have been gradually reduced in recent years. Chemotherapy is recognized as the mainstay of breast cancer treatment. However, this treatment usually has various degrees of side effects, resulting in a lot of distress in patients. Their original healthy lives were affected, which is characterized by disease and treatment. It was also reported that these patients had physical and mental health problems and a reduced quality of life in many ways [16]. According to surveys, the common symptoms of distress in breast cancer patients included abnormal defecation, insomnia, fatigue, and vision changes, which had an important impact on the survival and prognosis of patients [17, 18]. Domestic research on symptom distress in breast cancer patients is mainly focused on investigative research, and there are few clinical intervention trials at present. In recent years, the concept of breast cancer treatment has shifted from disease treatment to prognosis and rehabilitation. The goal of rehabilitation for breast cancer patients is to enable patients to obtain a full range of rehabilitation in appearance, function, employment, and psychology, etc.

In this study, symptom management theory was applied for nursing interventions in breast cancer patients. The results of this study showed that the symptom distress in the intervention group was significantly less than that in the control group. Moreover, the scores in terms of positive attitude, positive actions, close relationships, and total scores of hope levels were obviously higher than those in the control group, while the scores regarding physical well-being, social/family well-being, emotional well-being, functional well-being, additional concerns, and total scores of life quality were significantly increased, compared with those in the control group. In addition, in contrast to those in the control group, SAS scores, SDS scores, and VAS scores after intervention in the intervention group were remarkably decreased, while the PSQI scores in the intervention group were significantly increased. The above results indicated that nursing intervention based on symptom management theory could improve symptom distress, life quality, and sleep quality, as well as increase hope levels and reduce negative emotions and pain feelings. The results of this research were similar to those in the report by Houston [19]. Another study on the application of SMT-based palliative care in the interventional treatment of patients with advanced liver cancer found that the implementation of palliative care based on SMT could significantly alleviate cancer-related fatigue in these patients [20]. Hoffman reported that based on SMT, oncology nurses could have an obvious positive effect on the patients' lives through decreasing the symptom burden related to cancer and its treatment [21]. As we can see, the symptom management theory could understand the specific needs of nursing service in each patient according to the symptom assessment and was used to guide the nursing staff to implement individualized and targeted intervention measures so as to more effectively control the clinical symptoms of patients, promote their recovery, and make up for the lack of routine nursing care.

SMT provides a conceptual framework for understanding the factors that influence symptom perception and management. At the same time, it could also help hospital staff recognize the shortcomings and barriers in symptom management [22]. Many studies reported that SMT was considered as a useful framework for studying children with cancer and their parents [12, 23]. Another study analyzed and evaluated the SMT applicability in nursing care for pediatric oncology and other chronic diseases and demonstrated that SMT had the potential to guide nursing research and practice to improve symptoms in children with cancer [8]. Based on symptom management theory, this study paid attention to the occurrence of symptoms in breast cancer patients from emphasizing the perspective symptom clusters and the internal relationship between symptoms. This study also prevented the potential symptoms that may be caused by the current symptoms under the premise of effectively controlling the current symptoms themselves. The foreseeing implemented interventions were performed in this study, which effectively overcome the shortcomings of the present symptom management models [24]. In the process of intervening in breast cancer patients, the cognitive intervention method used in this study can be effective in improving the health status of patients because it can make patients aware of what symptoms are included in the chemotherapy symptom group, what symptoms they experience, what measures can be taken to prevent the onset of symptoms, and what measures can be taken to control or alleviate symptoms when they appear. The physical and psychological effects following chemotherapy underwent dynamic changes in breast cancer patients [25, 26]. By assessing the severity of the adverse symptoms, the nursing intervention plan based on SMT could provide personalized health management, fully arouse the enthusiasm of patients, and to the greatest extent, give patients' subjective initiative into full play. This nursing intervention plan also developed attainable goals and allowed the patient to reach them on their own. The hospital staff would assist when these patients encountered difficulties in the process of achieving their goals. It was indicated that the nursing intervention plan based on SMT was helpful in building the confidence of patients in self-management of symptoms [27, 28].

In conclusion, a nursing intervention plan based on symptom management theory meets the needs of breast cancer patients undergoing chemotherapy and could effectively improve symptom distress, increase hope levels, enhance life quality and sleep quality, relieve the pain degree, and decrease negative emotions, which are worth being promoted in clinical care. However, this study has some limitations, including being a single-center study, small sample size, short-term care interventions, and a lack of long-term follow-up results and categorical comparisons. Therefore, in order to draw more precise conclusions, we will conduct a multicenter randomized controlled trial with a larger sample size and conduct long-term follow-up.

## Figures and Tables

**Figure 1:** Comparison of SAS and SDS scores before and after intervention between the two groups. (a) SAS score. (b) SDS score. Compared with patients in the same group before intervention, ^*∗*^*P* < 0.05. Compared with patients in the control group after intervention, ^#^*P* < 0.05.

**Figure 2:** Comparison of VAS and PSQI scores before and after intervention between the two groups. (a) VAS score. (b) PSQI score. Compared with patients in the same group before intervention, ^*∗*^*P* < 0.05. Compared with patients in the control group after intervention, ^#^*P* < 0.05.

**Table 1:** The scores for the degree of severity of symptom clusters in patients with breast cancer.

Serial number	Symptom clusters	Average scores
1	Self-image damaged symptom clusters	2.60 ± 0.81
2	Perimenopausal symptom clusters	1.94 ± 0.75
3	Gastrointestinal symptom clusters	1.72 ± 0.82
4	Pain related symptom clusters	1.66 ± 0.71
5	Mental symptom clusters	1.45 ± 0.62
6	Nervous system related symptom clusters	1.39 ± 0.57

**Table 2:** Comparison of basic data between two groups.

Group	Control group (*n* = 60)	Intervention group (*n* = 60)	*χ * ^2^/*t* value	*P* value
Age (years)	42.5 ± 5.6	41.2 ± 5.5	1.283	0.202

Degree of education (n)			0.040	0.841
Below junior middle school	18	17		
Above junior middle school	42	43		

Duration of the disease (years)	3.8 ± 0.8	3.6 ± 0.7	1.457	0.148
BMI (kg/m^2^)	23.3 ± 1.6	23.7 ± 1.7	1.327	0.187

Neoplasm staging			1.682	0.641
I stage	10	11		
II stage	12	15		
III stage	33	32		
IV stage	5	2		

Marriage status (*n*)			1.362	0.506
Married	4	6		
Unmarried	42	36		
Widowed or divorced	14	18		

Health insurance (*n*)			0.536	0.464
Yes	55	57		
No	5	3		

On job (*n*)			0.574	0.449
Yes	20	24		
No	40	36		

Underlying disease (*n*)				
Hypertension	10	8	0.261	0.609
Diabetes	6	9	0.686	0.408

**Table 3:** Comparison of symptom distress before and after intervention between the two groups.

Groups	Cases (*n*)	Before intervention		After intervention	
		Symptom severity score	Symptom distress score	Symptom severity score	Symptom distress score
Control group	60	7.2 ± 2.2	8.2 ± 2.0	6.3 ± 2.0	6.4 ± 1.8
Intervention group	60	7.0 ± 2.4	8.0 ± 1.8	5.4 ± 2.1	5.5 ± 2.0
*t* value		0.475	0.575	2.403	2.590
*P* value		1.657	0.565	0.017	0.010

**Table 4:** Comparison of Herth Hope Index scores between the two groups.

Parameters	Before intervention					After intervention			
	Control group	Intervention group	*T* value	*P* value	Control group		Intervention group	*T* value	*P* value
Positive attitude	9.0 ± 1.2	9.3 ± 1.5	1.209	0.228	10.4 ± 1.5		12.2 ± 1.6	6.357	0.000
Positive actions	10.0 ± 1.5	10.2 ± 1.7	0.683	0.495	11.3 ± 2.0		12.3 ± 1.7	2.950	0.003
Close relationships	10.3 ± 2.0	10.4 ± 2.1	0.267	0.789	11.3 ± 1.7		12.1 ± 1.5	2.733	0.007
Total scores	29.3 ± 6.1	29.9 ± 6.4	0.525	0.600	33.0 ± 6.9		36.9 ± 5.6	3.399	0.000

**Table 5:** Comparison of life quality between two groups.

Parameters	Before intervention		*t* value	*P* value	After intervention		*t* value	*P* value
	Control group	Intervention group			Control group	Intervention group		
Physical well-being	2.5 ± 0.6	2.7 ± 0.6	1.825	0.070	3.2 ± 0.6	3.6 ± 0.5	3.967	<0.001
Social/family well-being	2.4 ± 0.7	2.6 ± 0.6	1.680	0.095	3.1 ± 0.6	3.5 ± 0.6	3.651	<0.001
Emotional well-being	2.5 ± 0.8	2.4 ± 0.7	0.728	0.467	3.2 ± 0.5	3.5 ± 0.6	2.975	0.003
Functional well-being	2.5 ± 0.7	2.3 ± 0.6	1.680	0.095	2.9 ± 0.6	3.3 ± 0.6	3.651	<0.001
Additional concerns	2.6 ± 0.6	2.7 ± 0.5	0.991	0.323	3.0 ± 0.4	3.4 ± 0.5	4.838	<0.001
Mean scores	2.5 ± 0.7	2.5 ± 0.6	0.000	1.000	3.1 ± 0.6	3.5 ± 0.5	3.967	<0.001

## Data Availability

The experimental data used to support the findings of this study are available from the corresponding author upon request.
